This article has been retracted.

# Hybrid Rider Optimization with Deep Learning Driven Biomedical Liver Cancer Detection and Classification

**DOI:** 10.1155/2022/6162445

**Published:** 2022-06-30

**Authors:** Mesfer Al Duhayyim, Hanan Abdullah Mengash, Radwa Marzouk, Mohamed K Nour, Hany Mahgoub, Fahd Althukair, Abdullah Mohamed

**Affiliations:** ^1^Department of Computer Science, College of Sciences and Humanities-Aflaj, Prince Sattam Bin Abdulaziz University, Al-Kharj, Saudi Arabia; ^2^Department of Information Systems, College of Computer and Information Sciences, Princess Nourah Bint Abdulrahman University, P.O. Box 84428, Riyadh 11671, Saudi Arabia; ^3^Department of Computer Sciences, College of Computing and Information System, Umm Al-Qura University, Mecca, Saudi Arabia; ^4^Department of Computer Science, College of Science & Art at Mahayel, King Khalid University, Abha, Saudi Arabia; ^5^Department of Computer Science, Faculty of Computers and Information, Menoufia University, Shibin Al Kawm, Egypt; ^6^Department of Electrical Engineering and Computer Sciences, College of Engineering, University of CA, Berkeley, USA; ^7^Research Center, Future University in Egypt, New Cairo 11845, Egypt

## Abstract

Biomedical engineering is the application of the principles and problem-solving methods of engineering to biology along with medicine. Computation intelligence is the study of design of intelligent agents which are systems acting perceptively. The computation intelligence paradigm offers more advantages to the enhancement and maintenance of the field of biomedical engineering. Liver cancer is the major reason of mortality worldwide. Earlier-stage diagnosis and treatment might increase the survival rate of liver cancer patients. Manual recognition of the cancer tissue is a time-consuming and difficult task. Hence, a computer-aided diagnosis (CAD) is employed in decision making procedures for accurate diagnosis and effective treatment. In contrast to classical image-dependent “semantic” feature evaluation from human expertise, deep learning techniques could learn feature representation automatically from sample images using convolutional neural network (CNN). This study introduces a Hybrid Rider Optimization with Deep Learning Driven Biomedical Liver Cancer Detection and Classification (HRO-DLBLCC) model. The proposed HRO-DLBLCC model majorly focuses on the identification of liver cancer in the medical images. To do so, the proposed HRO-DLBLCC model employs preprocessing in two stages, namely, Gabor filtering (GF) based noise removal and watershed transform based segmentation. In addition, the proposed HRO-DLBLCC model involves NAdam optimizer with DenseNet-201 based feature extractor to generate an optimal set of feature vectors. Finally, the HRO algorithm with recurrent neural network–long short-term memory (RNN-LSTM) model is applied for liver cancer classification, in which the hyperparameters of the RNN-LSTM model are tuned by the use of HRO algorithm. The HRO-DLBLCC model is experimentally validated and compared with existing models. The experimental results assured the promising performance of the HRO-DLBLCC model over recent approaches.

## 1. Introduction

Liver disease is one of the severe medical states which may threaten human health and life. Liver tumors are considered the second main cause of mortality rates in males and the sixth main reason of mortality rates in women. In 2008, 7,50,000 individuals were found to have liver malevolence and 9,60,000 individuals deceased because of this disease [1]. CT scan is considered a famous method for surgical scheduling and prognosis of body parts in the abdomen region [2]. Thus, CT scan is frequently utilized for diagnosing liver cancer. Liver division is a crucial stage in computer-aided therapeutic interpolation by utilizing CT images like radiation, surgery of liver transplantation, and volume estimation. Physical allotment of every slice is an ordinary medical trial for the liver description. So, manual segmentation is time-consuming, ineffective, and autonomous. In this way, for designing a fully mechanical system with monitoring, expediting, and diagnosing ability, therapeutic planning is crucial. Several methods to segment the liver in CT scans were explained, and an overview of such methods is given in [3]. Usually, such methodologies are categorized into 3 groups: automatic, interactive, and semiautomatic [4].

Semiautomatic and interactive methodologies rely on little or huge user communication whereas automatic methodologies do not rely on any kind of user communication [5]. Semiautomatic methods have a capability to diminish the efficiency of a doctor. For effective classification of liver cancer, artificial intelligence (AI) and image processing methods have an ability in research applications [6]. Various approaches to identifying liver tumor are announced, involving region oriented methodologies, machine learning (ML), and watershed transform method. Deep learning (DL) is generally an easier route for normalizing the picture element of an image to the equal level [7]. The images, which are thus extracted, may imitate the characteristics of the images for preprocessed images; the state of the derived characteristics denotes the correctness of the role importantly [8]. At last, a conclusion that the object group in the picture is the core component of DL has been made, and this becomes a matter of major current works. ML method has attained superior radiological efficacy and might solve this break in the radiological categorization of distinct syndromes [9]. FCNNs (fully convolutional neural networks) do not require explanation of some radiological characteristics for recognizing images, and, in contrast to other ML methods, they might also find some characteristics which are not available in today's radiological practices [10].

This study introduces a Hybrid Rider Optimization with Deep Learning Driven Biomedical Liver Cancer Detection and Classification (HRO-DLBLCC) model. The proposed HRO-DLBLCC model employs preprocessing in 2 stages, namely, Gabor filtering (GF) related noise removal and watershed transform based segmentation. In addition, the proposed HRO-DLBLCC model involves NAdam optimizer with DenseNet-201 based feature extractor to generate an optimal set of feature vectors. Finally, the HRO algorithm with recurrent neural network–long short-term memory (RNN-LSTM) methodology is applied for liver cancer classification. The HRO-DLBLCC model is experimentally validated and compared with existing models.

## 2. Related Works

This section offers a detailed review of liver cancer detection and classification models. In [11], an innovative approach which focuses on eliminating the essential data to the least feasible set of circulating miRNAs is suggested. The dimensional diminution reached imitates a highly significant stage in clinically actionable, potential, circulating miRNA related accuracy medicine pipelines. Heterogeneous ensembles could reimburse intrinsic prejudices of classifiers by utilizing distinct classifier methods. Sadeque et al. [12] introduce an automatic methodology of identifying liver cancer in abdominal CT images and categorizing them with the help of the histogram of an oriented gradient-support vector machine (HOG-SVM). The image segmentation and liver region abstraction are carried out in the subsequent step compiling contouring and thresholding. We compiled ROI related histogram oriented gradient (HOG) feature extraction for training the classifier that urges the classifier to be quicker than the traditional methodologies.

Randhawa et al. [13] suggested a hybrid method that blends the regularization operation with the recent loss function for the support vector machine (SVM) categorization. The gray level cooccurrence matrix (GLCM) has been executed to derive the characteristics from the image. The derived characteristics which nourished to SVM classifier are extracted by utilizing selected feature vectors for categorizing the influenced area and ignoring the unnecessary regions. In [14], the researchers suggest an analysis of an original 3D-CNN devised for tissue categorization in medicinal imaging and applied for differentiating metastatic liver and primary tumors from distribution weight MRI (DW-MRI) information. The suggested network is made up of 4 sequential stridden 3D convolution layers with 3 × 3 × 3 kernel size and ReLU as activation operation, succeeded by whole connected layers with 2,048 neurons and softmax layers for a dual classifier.

In [15], an automated CAD structure is provided in 3 levels. The first level is automated liver separation, and lesion identification of lesion is performed. The second level is extracting characteristics. Finally, liver lesion categorization into benign and malignant is made with the help of the original contrast related feature difference methodology. The features which are extracted from the lesion region having its surrounding normal liver tissue depend on texture and intensity. The lesion descriptor is attained by assuming the distinction between the characteristics of normal tissue and those of lesion region of liver. At last, for classifying the liver lesions into benign or malignant, a new SVM related machine learning (ML) classifier is trained on the new descriptors. Moorthi and Agita [16] suggested a fresh technique termed Level Set-related Back Propagation Neural Network (LS-BPNN) for the mechanical classification and recognition of liver cancer. In [17–20], the researchers enhanced a DL oriented assistant for helping diagnosticians distinguish between 2 sub-kinds of fundamental liver cancer, cholangiocarcinoma and hepatocellular carcinoma, on eosin and hematoxylin stained whole slide images (WSI) and assessed its impact on the diagnostic outcomes of eleven diagnosticians with changing stages of skills.

Several CAD models exist in the literature to classify the presence of liver cancer using medical images. Though several ML and DL models for liver cancer classification are available in the literature, enhancement of the classification performance is still needed. Owing to continual deepening of the DL model, the number of its parameters also increases quickly, which results in model overfitting. At the same time, different hyperparameters have a significant impact on the efficiency of the CNN model. Particularly, hyperparameters such as epoch count, batch size, and learning rate selection are essential to attain effectual outcome. Since the trial and error method for hyperparameter tuning is a tedious and erroneous process, metaheuristic algorithms can be applied. Therefore, in this work, we employ HRO algorithm for the parameter selection of the RNN-LSTM model.

## 3. The Proposed Model

In this study, a new HRO-DLBLCC method was enhanced for the effectual identification of liver cancer in the medical images. The proposed HRO-DLBLCC model employed preprocessing in two stages, namely, GF based noise removal and watershed transform based segmentation. NAdam optimizer with DenseNet-201-based feature extractor, RNN-LSTM-based liver cancer classifier, and HRO-related hyperparameter tuning.  Figure 1 illustrates the block diagram of HRO-DLBLCC approach.

### 3.1. Image Preprocessing

At the primary stage, the suggested HRO-DLBLCC method employed preprocessing in 2 stages, namely, GF related noise removal and watershed transform based segmentation. The GF technique has two mechanisms known as sinusoidal and Gaussian. This component can link the optimum representation of the orientation direction and the spatial domain [21]. The GF of the image is mathematically expressed in the following equation, where the cosine wave frequency can be represented as *fr*, *u*, and *v* axes; *σ*_*u*_ and *σ*_*v*_ refer to the fixed distance from the Gaussian property; and *θ* indicates the orientation direction. Furthermore, *u*_*θ*_ and *v*_*θ*_ representations are shown in (2) and (3), respectively:

(1) $$\begin{array}{c} GF\left(u,v;\theta ,fr\right)=\text{exp}\left\{-\frac{1}{2}\left[\frac{u_{\theta \prime }^{2}}{\sigma_{u}^{2}}+\frac{v_{\theta }^{2}}{\sigma_{v}^{2}}\right]\right\}\text{cos}\left(2\Pi fru_{\theta }\right), \end{array}$$

(2) $$\begin{array}{c} u_{\theta }=u\text{cos}\theta -v\text{sin}\theta , \end{array}$$

(3) $$\begin{array}{c} v_{\theta }=u\text{sin}\theta +v\text{cos}\theta . \end{array}$$

Then, the watershed transform model is employed for image segmentation. This region related segmentation model works on the principle of geography. Here, the grayscale image is considered a topographic relief and has a local minimum called a catchment basin. Once the water is submerged, it constructs a barrier and constitutes a watershed. This methodology produces overall division of an image. The morphological process is utilized for attaining structure of an image. In general, this process suppresses noise of the system and other artefacts from the greyscale images. Then, the presented model is applied to the gradient images for smooth structure of the boundary.

### 3.2. Feature Extraction

Next to image preprocessing, the DenseNet-201 based feature extractor generates an optimal set of feature vectors. The DenseNet-201 exploits condensed network which provides efficiency and simple training as a result of the potential feature applied for different layers, which increases the variance in the following layer, thereby improving the performance of the system. This architecture showcases typical functions under various datasets such as CIFAR-100 and ImageNet. The improved connectivity in a DenseNet-201 system and the direct communication between a layer and the following layers are deployed as demonstrated in Figure 2.

(4) $$\begin{array}{c} z^{l}=H_{l}\left(\left[z^{0},z^{1},\ldots \ldots ,z^{l-1}\right]\right). \end{array}$$

In (4), *H*_*l*_ means a nonlinear transform that is defined by a composite function using BN, ReLU, and a Conv of 3 × 3. [*z*^0^, *z*^1^,……, *z*^*l*−1^] showcases a feature map combination of layers from the resultant layer 0 to *l* − 1 that is incorporated into a tensor for easier execution. For the downsampling model, dense block is improved for isolation, and transition layers have BN with 2 × 2 average pooling layer and 1 × 1 Conv layer. The progressive rate in DenseNet-201 describes how dense architecture achieves new intention to hyperparameter *k*. It calculates the progression rate where the feature map is regarded as the global state. Therefore, a consecutive layer is comprised of feature map with the preceding layer. *k* feature map is added to the global state by all the layers whereby total input feature maps at *l*^*th*^ layers (*FM*)^*l*^ are shown as follows:

(5) $$\begin{array}{c} {\left(FM\right)}^{l}=k^{0}+k\left(l-1\right). \end{array}$$

In (5), channel in an input layer is denoted by *k*^0^. To increase the processing effectiveness, a 1 × 1 Conv layer was deployed for each 3 × 3 Conv layer that mitigates the total volume of input feature maps, namely, greater than that of *k* output feature map. Therefore, the 1 × 1 Conv layer is known as the bottleneck layer, and it generates 4*k* feature maps.

For classification purposes [22], 2 dense layers with neurons are enclosed. The feature extraction with sigmoid activation function and DenseNet-201 is used for calculating dual classifications, with softmax activation function used as conventional DenseNet-201 architecture. A neuron existing in the FC dense layer is interconnected to all neurons in the prior layer. It is numerically determined as FC layer 1 in which input 2  *D* feature map is expanded for 1  *D* feature vector:

(6) $$\begin{array}{c} t^{l-1}=\text{Bernoulli}\left(p\right),\\ {\ddot{x}}^{l-1}=t^{l-1}*c^{l-1},\\ {\ddot{x}}^{l}=f\left(w^{k}{\ddot{x}}^{l-1}+o^{l}\right). \end{array}$$

The Bernoulli function generates a vector *t*^*l*−1^ arbitrarily by probability of concerning 0-1 distribution. *c*^*l*−1^ characterizes the vector dimension. In 2 layers of the FC, layer employs a dropout principle for blocking certain neurons on the basis of the desired probability that prevents overfitting problems. *w*^*l*^ and *o*^*l*^ define the weight along with offset variable of the FC layer. A sigmoid activation function is used for altering non-normalized outcomes into binary output as one or zero.

The proposed HRO-DLBLCC model involves NAdam optimizer for hyperparameter tuning of the DenseNet-201 model. The NAdam optimizer attempted to incorporate Nesterov's accelerated adaptive moment estimation within Adam. A substantial benefit of this integration method is that adaptive moment estimation assists in executing different phases in a gradient fashion by upgrading variables with momentum stage before the gradient calculation. The upgrade rule of NAdam is illustrated as follows:

(7) $$\begin{array}{c} w_{t}=w_{t-1}-\alpha \times \frac{{\bar{m}}_{t}}{\sqrt{{\hat{v}}_{t}}+\varepsilon }, \end{array}$$

But

(8) $$\begin{array}{c} {\bar{m}}_{t}=\left(1-\beta_{1,t}\right){\hat{g}}_{t}+\beta_{1,t+1}{\hat{m}}_{t},\\ {\hat{m}}_{t}=\frac{m_{t}}{1-\prod_{i=1}^{t+1}\beta_{1i}},\\ {\hat{g}}_{t}=\frac{g_{t}}{1-\prod_{i=1}^{t+1}\beta_{1i}}. \end{array}$$

### 3.3. RNN-LSTM Based Image Classification

Once the features are generated, the RNN-LSTM model is utilized for the detection and classification of liver cancer. The recurrent NN is comprised of long-term memory through weights. It can be different in training duration and encode the comprehensive knowledge regarding the dataset. Furthermore, short-term memory in terms of ephemeral function is passed from individual to following nodes [23]. In this model, LSTM method indicates an intermediate type of memory cell. The unit of LSTM cell is described and enumerated. For instance, *s* denotes a vector with measure of *s*_*c*_ at every memory cell *c*. Once *c* subscript is employed, it helps in an individual memory cell. Generally, the input node is named *g*. Now, gates are called  *y*_*in*_ and *y*_*out*_; however, the conflict of *y*  shows an improved outcome in the ML method. Furthermore, it employs *u*,  *f*, and *o* to determine outcome, input, and forget gates.

The peephole relationships handed from inner state to output and input gates of the similar node lack most important rules to be employed in output gate. Assume a system that evaluates objects and produces essential outcomes while *n*  objects are regarded. In addition, the scheme recognizes dissimilar amounts of activation to the inner state. This activation has appeared in the inner state *s*_*c*_ with constant error container and improved. Once *n*th object is deliberated, the system needs to discover the inner state. It can be achieved through output gates *o*_*c*_ to acquire the substantial formula of inner state *s*_*c*_. Hence, *s*_*c*_ must be input to *o*_*c*_. The approximation of LSTM depends on memory cells properly. The successive procedure is executed for each iteration. The expression employed for current LSTM using forget gate is represented as follows:

(9) $$\begin{array}{c} g^{\left(z\right)}=\varphi \left(W^{gl}l^{\left(z\right)}+W^{gh}h^{\left(z-1\right)}+b_{g}\right),\\ u^{\left(z\right)}=\sigma \left(W^{ul}l^{\left(t\right)}+W^{uh}h^{\left(z-1\right)}+b_{u}\right),\\ f^{\left(z\right)}=\sigma \left(W^{fl}l^{\left(t\right)}+W^{fh}h^{\left(z-1\right)}+b_{f}\right),\\ o^{\left(z\right)}=\sigma \left(W^{ol}l^{\left(t\right)}+W^{oh}h^{\left(z-1\right)}+b_{o}\right),\\ s^{\left(z\right)}=\;g^{\left(z\right)}⊙u^{\left(u\right)}+s^{\left(z-1\right)}⊙f^{\left(t\right)},\\ h^{\left(z\right)}=\phi \left(s^{\left(z\right)}\right)⊙o^{\left(t\right)}. \end{array}$$

The measures of hidden state of LSTM at time *z* are portrayed as vector *h*^(*z*)^, as *h*^(*z* − 1)^ describes the amount of memory cells in hidden state at prior time. Consider the forget gate, the peephole connection is not present. The process becomes simpler for LSTM without forget gate and is achieved by *f*^(*z*)^=1 to all  *z*. At the same time, using a forward pass, LSTM is induced for inner state. It is assumed that input gate has achieved value of 0, and no activation function can be obtained. Then, LSTM has executed maximal capability for understanding longer range dependency as applicable for simple RNN.

### 3.4. Hyperparameter Optimization

In the final stage, the hyperparameter optimization of the RNN-LSTM model is performed by the use of HRO algorithm. The HRO algorithm is derived by the fusion of rider optimization algorithm (ROA) and sunflower optimization (SFO). There are four dissimilar kinds of riders, namely, attacker, bypass rider, overtaker, and follower. ROA works by the behavior of dissimilar kinds of rider to the termination [24]. The SFO works by the revolution of sun. Sunflower often imitates the revolution that is naturally inspired by optimization. This mechanism could define a better location for effective outcome. Simultaneously, it makes use of higher computational difficulty as a result of higher computational steps. To attain an optimal global solution with fast performance and better computational steps, we employ hybrid ROA approach with the SFO. At the first level, parameter initialization process is carried out. For updating location, we employ bypass rider to increase the accomplishment rate. Bypass riders frequently follow and track a route without rider information. The formula for updating location according to the bypass rider is represented as follows:

(10) $$\begin{array}{c} B_{t+1}\left(r,p\right)=\partial \left[B_{t}\left(t,p\right)*m\left(p\right)+B_{t}\left(\mu ,p\right)*\left[1-m\left(p\right)\right]\right]. \end{array}$$

Here, the variables *∂*, *t*, *m*, and *μ* specify the arbitrary amounts within [0,1] and *k* denotes the iteration number, which is determined by the user. Assume that *μ*=*r*; the formula can be expressed as follows:

(11) $$\begin{array}{c} B_{t+1}\left(r,p\right)=\partial \left[B_{t}\left(t,\;p\right)*m\left(p\right)+B_{t}\left(r,p\right)*\left[1-m\left(p\right)\right]\right]. \end{array}$$

The SFO updates the location or solution space through the revolution of sun. Sunflower often imitates the revolution of sun. Therefore, the location updating of SFO is represented as follows:

(12) $$\begin{array}{c} B\left(r,p\right)=B_{t}\left(r,p\right)+y_{r}\times g_{r}. \end{array}$$

In (12), *B*_*r*_(*r*,  *p*) represents the existing location at *t* time, *B*_*r*+1_(*r*,  *p*) indicates the upgraded location at *t* +1 time, *B*_*t*+1_(*r*, *p*) signifies the steps of sunflower, and *g*_*r*_ stands for the sunflower direction.

(13) $$\begin{array}{c} B_{t}\left(r,p\right)=\frac{B_{t+1}\left(r,p\right)}{y_{r}}\times g_{r}. \end{array}$$

For updating location, replace (14) which is the updating location of SFO in (12) which is the updating location of ROA.

(14) $$\begin{array}{c} B_{t+1}\left(r,p\right)=\partial B_{t}\left(t,p\right)*m\left(p\right)+\left(\frac{B_{t+1}\left(r,p\right)}{y_{r}}\right)\times g_{r}*\left[1-m\left(p\right)\right], \end{array}$$

(15) $$\begin{array}{c} B_{t+1}\left(r,p\right)=\partial B_{t}\left(t,p\right)*m\left(p\right)+B_{t+1}\left(r,p\right)\left[1-m\left(p\right)\right]-y_{r}\times g_{r}*\left[1-m\left(p\right)\right]. \end{array}$$

Later, rearranging (16) and (17), we acquire

(16) $$\begin{array}{c} B_{t+1}\left(r,p\right)=\partial B_{t}\left(t,p\right)*m\left(p\right)+B_{t+1}\left(r,p\right)-\frac{B_{t+1}\left(r,p\right)m\left(p\right)}{y_{r}g_{r}}+y_{r}g_{r}m\left(p\right),\\ \frac{B_{t+1}\left(r,p\right)}{B_{t+1}\left(r,p\right)\partial }+\partial B_{r+1}\left(r,p\right)m\left(p\right)=\partial \left[\frac{B_{t}\left(t,p\right)*m\left(p\right)}{y_{r}t_{r}+y_{r}t_{r}m\left(p\right)}\right],\\ B_{t+1}\left(r,p\right)\left[1-\partial +\partial m\left(p\right)\right]=\partial \left[\frac{B_{t}\left(t,p\right)*m\left(p\right)}{y_{r}t_{r}+y_{r}t_{r}m\left(p\right)}\right]. \end{array}$$

Next, the last formula can be expressed as follows:

(17) $$\begin{array}{c} Bt+1\left(r,p\right)=\frac{1}{\left[1-\partial \left[1-m\left(p\right)\right]\right]}\left[\frac{\partial \left[Bt\left(t,p\right)*m\left(p\right)\right]}{y_{r}t_{r}\left[1-m\left(p\right)\right]}\right]. \end{array}$$

At present, the highest fitness values are regarded as an optimal solution, and ROA variables are updated for the optimal solution. The abovementioned steps are iterated until the iteration amount is attained. The HRO approach extracts a fitness function for obtaining enhanced classifier performances. It fixes a positive integer to indicate the superior execution of the applicant solutions. In this article, the reduction of the classifier fault rate is regarded as the fitness function, as provided in (18). The optimum resolution contains a minimum fault rate, and the poor solution gets an inclined error rate.

(18) $$\begin{array}{c} \text{fitness}\left(x_{i}\right)=\text{ClassifierErrorRate}\left(x_{i}\right)=\frac{\text{number of misclassified samples}}{\text{Total number of samples}}*100. \end{array}$$

## 4. Experimental Validation

This section examines the liver cancer classification results of the HRO-DLBLCC model using a set of medical images. The proposed model is simulated using Python 3.6.5 tool. The dataset holds a total of 1500 images with three classes, namely, hemangioma (HEM), hepatocellular carcinoma (HCC), and metastatic carcinoma (MET). The details related to the dataset are given in Table 1. A few sample images are shown in Figure 3.

Figure 4 highlights the confusion matrices created by the HRO-DLBLCC model on the test data. With entire dataset, the HRO-DLBLCC model has categorized 497 samples as HEM class, 497 samples as HCC class, and 483 samples as MET class. Moreover, with 70% of TR data, the HRO-DLBLCC method has categorized 357 samples as HEM class, 344 samples as HCC class, and 322 samples as MET class. Besides, with 30% of TS data, the HRO-DLBLCC technique has categorized 140 samples as HEM class, 153 samples as HCC class, and 151 samples as MET class.

Table 2offers a comprehensive liver cancer classification result of the HRO-DLBLCC model.  Figure 5 exhibits a brief classifier result of the HRO-DLBLCC model on the entire dataset. The results indicated that the HRO-DLBLCC model has recognized all the classes effectively on the entire dataset. For instance, the HRO-DLBLCC model has recognized samples under HEM class with *accu*_*y*_, *prec*_*n*_, *reca*_*l*_, *F*_score_, and MCC of 99%, 97.64%, 99.40%, 98.51%, and 97.77%, respectively.

Additionally, the HRO-DLBLCC methodology has recognized samples under HCC class with *accu*_*y*_, *prec*_*n*_, *reca*_*l*_, *F*_score_, and MCC of 99.33%, 98.61%, 99.40%, 99%, and 98.50%, respectively. Besides, the HRO-DLBLCC algorithm has recognized samples under MET class with *accu*_*y*_, *prec*_*n*_, *reca*_*l*_, *F*_score_, and MCC of 98.60%, 99.18%, 96.60%, 97.87%, and 96.85%, respectively.

Figure 6 displays a brief classifier outcome of the HRO-DLBLCC algorithm on the 70% of TR dataset. The results specified that the HRO-DLBLCC technique has recognized all the classes effectively on the entire dataset. For example, the HRO-DLBLCC model has recognized samples under HEM class with *accu*_*y*_, *prec*_*n*_, *reca*_*l*_, *F*_*score*_, and MCC of 99.05%, 97.81%, 99.44%, 98.62%, and 97.90%, respectively. In addition, the HRO-DLBLCC approach has recognized samples under HCC class with *accu*_*y*_, *prec*_*n*_, *reca*_*l*_, *F*_score_, and MCC of 99.14%, 98.01%, 99.42%, 98.71%, and 98.07%, respectively. Besides, the HRO-DLBLCC model has recognized samples under MET class with *accu*_*y*_, *prec*_*n*_, *reca*_*l*_, *F*_score_, and MCC of 98.57%, 99.40%, 96.23%, 97.79%, and 96.76%, respectively.

Figure 7 shows a brief classifier outcome of the HRO-DLBLCC methodology on 30% of the TS data. The results specified that the HRO-DLBLCC model has recognized all the classes effectively on the entire dataset. For example, the HRO-DLBLCC algorithm has recognized samples under HEM class with *accu*_*y*_, *prec*_*n*_, *reca*_*l*_, *F*_score_, and MCC of 98.89%, 97.22%, 99.29%, 98.25%, and 97.44%, respectively. Moreover, the HRO-DLBLCC technique has recognized samples under HCC class with *accu*_*y*_, *prec*_*n*_, *reca*_*l*_, *F*_score_, and MCC of 99.78%, 100%, 99.35%, 99.67%, and 99.51%, respectively. Furthermore, the HRO-DLBLCC techniques have recognized samples under MET class with *accu*_*y*_, *prec*_*n*_, *reca*_*l*_, *F*_score_, and MCC of 98.67%, 98.69%, 97.42%, 98.05%, and 97.04%, respectively.

The training accuracy (TA) and validation accuracy (VA) attained by the HRO-DLBLCC system on the test dataset are demonstrated in Figure 8. The experimental outcome implied that the HRO-DLBLCC approach has gained maximum values of TA and VA. Specifically, the VA seemed to be superior to TA.

The training loss (TL) and validation loss (VL) achieved by the HRO-DLBLCC algorithm on the test dataset are established in Figure 9. The experimental outcome inferred that the HRO-DLBLCC methodology has accomplished least values of TL and VL. Specifically, the VL seemed lower than TL.

A brief precision-recall examination of the HRO-DLBLCC model on the test dataset is shown in Figure 10. By observing the figure, it can be noticed that the HRO-DLBLCC method has accomplished maximal precision-recall performance under all classes.

A detailed ROC investigation of the HRO-DLBLCC approach on the test dataset is represented in Figure 11. The results indicated that the HRO-DLBLCC model has exhibited its ability to categorize three different classes, namely, HEM, HCC, and MET, on the test dataset.

In order to report the enhanced performance of the HRO-DLBLCC model, a wide-ranging comparative study is made in Table 3 [25, 26].  Figure 12 illustrates a comparative *accu*_*y*_ examination of the HRO-DLBLCC model with recent models. The figure indicates that the AdaBoost, NB, and MLP models have shown lower *accu*_*y*_ values of 90.96%, 91.41%, and 91.93%, respectively. At the same time, the KNN model has exhibited slightly improved *accu*_*y*_ of 93.79%. It is followed by the SVM, J48, and RF models which have demonstrated closer *accu*_*y*_ values of 95.77%, 96.43%, and 95.24%, respectively. However, the HRO-DLBLCC model has surpassed all other models with maximum *accu*_*y*_ of 99.11%.

Figure 13 demonstrates a comparative *prec*_*n*_ inspection of the HRO-DLBLCC method with recent models. The figure specifies that the AdaBoost, NB, and MLP techniques have shown lower *prec*_*n*_ values of 92.08%, 93.32%, and 92.76%, respectively. Meanwhile, the KNN approach has shown slightly enhanced *prec*_*n*_ of 95.65%. Next, the SVM, J48, and RF models have established closer *prec*_*n*_ values of 95.12%, 97.04%, and 94.97%, respectively. However, the HRO-DLBLCC method has surpassed all other models with maximal *prec*_*n*_ of 98.64%.

Figure 14 demonstrates a comparative *reca*_*l*_ inspection of the HRO-DLBLCC methodology with recent models. The figure indicates that the AdaBoost, NB, and MLP methodologies have shown reduced *reca*_*l*_ values of 87.99%, 89.49%, and 89.63%, respectively. Meanwhile, the KNN model has displayed slightly improved *reca*_*l*_ of 92.49%. It is followed by the SVM, J48, and RF techniques which have demonstrated closer *reca*_*l*_ values of 93.71%, 95.30%, and 94.47%, respectively. But the HRO-DLBLCC approach has surpassed all other techniques with maximal *reca*_*l*_ of 98.69%.

Figure 15 depicts a comparative *F*_score_ analysis of the HRO-DLBLCC technique with recent algorithms. The figure indicates that the AdaBoost, NB, and MLP models have shown lower *F*_score_ values of 89.72%, 89.50%, and 91.17%, respectively. Besides, the KNN model has exhibited slightly improved *F*_score_ of 89.68%, followed by the SVM, J48, and RF approaches which have demonstrated closer *F*_score_ values of 91.17%, 94.09%, and 95.57%, respectively. At last, the HRO-DLBLCC technique has surpassed all other techniques with maximal *F*_score_ of 98.66%.

From the detailed results and discussion, it is ensured that the HRO-DLBLCC model has accomplished maximum liver cancer classification outcomes.

## 5. Conclusion

In this study, a new HRO-DLBLCC method was enhanced for the effectual identification of liver cancer in medical images. The proposed HRO-DLBLCC model follows different stages, such as GF based noise removal, watershed segmentation, NAdam optimizer with DenseNet-201 based feature extractor, RNN-LSTM classification, and HRO based parameter tuning. The HRO-DLBLCC model is experimentally validated and compared with existing models. The experimental outcome ensured the promising performance of the HRO-DLBLCC model over recent approaches with maximum accuracy of 99.11%. In the future, the classification performance of the HRO-DLBLCC model can be improved by the use of deep instance segmentation approaches. In addition, the proposed model can be extended to the design of multimodal fusion based DL models to attain improved classification results.

## Figures and Tables

**Figure 1:** Block diagram of HRO-DLBLCC technique.

**Figure 2:** Layered structure in DenseNet-201.

**Figure 3:** Sample images.

**Figure 4:** Confusion matrices of HRO-DLBLCC technique: (a) entire dataset, (b) 70% of TR data, and (c) 30% of TS data.

**Figure 5:** Result analysis of HRO-DLBLCC algorithm under entire dataset.

**Figure 6:** Result analysis of HRO-DLBLCC algorithm under 70% of TR data.

**Figure 7:** Result analysis of HRO-DLBLCC algorithm under 30% of TS data.

**Figure 8:** TA and VA analysis of HRO-DLBLCC algorithm.

**Figure 9:** TL and VL analysis of HRO-DLBLCC algorithm.

**Figure 10:** Precision-recall curve analysis of HRO-DLBLCC algorithm.

**Figure 11:** ROC curve analysis of HRO-DLBLCC algorithm.

**Figure 12:** *Accu*_*y*_ analysis of HRO-DLBLCC algorithms with existing methodologies.

**Figure 13:** *prec*_*n*_ analysis of HRO-DLBLCC algorithms with existing methodologies.

**Figure 14:** Re*ca*_*l*_ analysis of HRO-DLBLCC algorithms with existing methodologies.

**Figure 15:** *F*_score_ analysis of HRO-DLBLCC algorithms with existing methodologies.

**Table 1:** Dataset details.

Label	Class names	No. of images
HEM	Hemangioma	500
HCC	Hepatocellular carcinoma	500
MET	Metastatic carcinoma	500
Total no. of images		1500

**Table 2:** Result analysis of HRO-DLBLCC technique with various measures.

Label	Accuracy	Precision	Recall	F-score	MCC
*Entire dataset*					
HEM	99.00	97.64	99.40	98.51	97.77
HCC	99.33	98.61	99.40	99.00	98.50
MET	98.60	99.18	96.60	97.87	96.85
Average	**98.98**	**98.48**	**98.47**	**98.46**	**97.71**

*Training phase (70%)*					
HEM	99.05	97.81	99.44	98.62	97.90
HCC	99.14	98.01	99.42	98.71	98.07
MET	98.57	99.40	96.23	97.79	96.76
Average	**98.92**	**98.41**	**98.37**	**98.37**	**97.58**

*Testing phase (30%)*					
HEM	98.89	97.22	99.29	98.25	97.44
HCC	99.78	100.00	99.35	99.67	99.51
MET	98.67	98.69	97.42	98.05	97.04
Average	**99.11**	**98.64**	**98.69**	**98.66**	**98.00**

**Table 3:** Comparative analysis of HRO-DLBLCC technique with existing algorithms.

Methods	Accuracy	Precision	Recall	F-score
Naïve Bayes	91.41	93.32	89.49	89.50
MLP algorithm	91.93	92.76	89.63	91.17
SVM algorithm	95.77	95.12	93.71	91.17
KNN algorithm	93.79	95.65	92.49	89.68
AdaBoost	90.96	92.08	87.99	89.72
J48 algorithm	96.43	97.04	95.30	94.09
Random forest	95.24	94.97	94.47	95.57
HRO-DLBLCC	99.11	98.64	98.69	98.66

## Data Availability

Data sharing is not applicable to this article as no datasets were generated during the current study.
